# Trends and barriers of emergency medical service use in Addis Ababa; Ethiopia

**DOI:** 10.1186/s12873-019-0242-5

**Published:** 2019-04-18

**Authors:** Menbeu Sultan, Yonas Abebe, Assefu Welde Tsadik, Asmamaw Ababa, Alegnta Gebre Yesus, Nee-Kofi Mould-Millman

**Affiliations:** 1 Department of Emergency Medicine and Critical Care, St. Paul’s Hospital Millennium Medical College, Addis Ababa, Ethiopia; 2 Department of Emergency Medicine and Critical Care nursing, St. Paul’s Hospital Millennium Medical College, Addis Ababa, Ethiopia; 3 Ethiopian Federal Ministry of Health, Emergency and Critical Care Directorate, Addis Ababa, Ethiopia; 4 Department of Emergency Medicine and Critical Care, Addis Ababa University School of Medicine, Addis Ababa, Ethiopia; 5 University of Colorado School of Medicine, Aurora, USA

**Keywords:** EMS, Use, Barriers, Ambulance, Language, Addis Ababa

## Abstract

**Background:**

The increasing burdens of trauma and time sensitive non-communicable disease in Addis Ababa necessitate a robust emergency medical care system. The objectives of this study were to assess the proportion of patients who used emergency medical services (EMS) and to quantitatively and qualitatively assess barriers to EMS utilization in Addis Ababa.

**Methods:**

A cross-sectional quantitative and qualitative study was conducted on patients who visited five selected public hospitals in Addis Ababa with specific emergency conditions. Data were collected by trained nurses using a standardized questionnaire. Descriptive statistics and logistic regression was done on cleaned and coded quantitative data using SPSS version 20. Thematic analysis was performed on the qualitative data. Ethical approval was obtained prior to the study.

**Results:**

A total of 429 participants completed the survey with a non-response rate of 5.1%. The most common emergency scene was the home (*n* = 222, 51.8%) followed by road side (*n* = 159, 37.1%). Only 87(20.3%) patients arrived by ambulance, though a majority (53.4%) of participants recalled at least one access number for an ambulance service and 96.3% stated that ambulances were an important part of the continuum of care for their emergency condition. A higher proportion of participants believed that ambulance transportation is generally safer (*n* = 341, 78.5%) and faster (*n* = 298, 69.5%) than emergency transport by taxi or private car. Patients who were non-Amharic speaking had a negative association with arriving by ambulance (*P* = 0.001, OR 0.47; C.I, 0.31, 0.71). The median acceptable time to get the ambulance (according to respondent’s perception) was 16 min but actually perceived ambulance waiting time was 40 min.

**Conclusion:**

EMS utilization in Addis Ababa is relatively low and emergency patients are instead being transported by taxi or private car. Perceived longer ambulance waiting time and language barriers may have contributed for low utilization. Findings of this study suggest an action to improve access by improving ambulance availability while simultaneously enhancing the public’s knowledge and perception of EMS in Addis Ababa.

## Background

Emergency medical services(EMS) systems are reported to be effective public health intervention to reduce mortality related to injuries and acute medical illnesses [1]. According to the world health organization, the majority of trauma related deaths occur in the pre-hospital setting. Ethiopia has amongst the highest road fatality rates in Africa with 68 fatalities per 10,000 vehicles per year. Furthermore, 28% of emergency room visits in Ethiopia are related to trauma, which predominantly affects a younger and economically productive socio demographic group [2]. In addition, non-communicable diseases are increasing; cardiovascular disease accounts for 24% of adult deaths [3, 4]. The high burden of trauma and acute illnesses, coupled with the increasing elderly population in Addis Ababa, demands improved access to an EMS system.

In-hospital and pre-hospital emergency care have experienced dramatic development in Addis Ababa over the past decade. Emergency rooms are being staffed by emergency specialist doctors and nurses. Advanced trauma care providers and specialty centers, including cardiac and trauma care, are increasing in number. But, it is reported that emergency patients are arriving to the treatment centers too late; after the golden hour has already passed or having already developed complications [5, 6].

Addis Ababa Fire and Emergency Prevention and Control Authority (AAFEPCA), along with a few private companies, provide the major pre-hospital emergency services throughout the city. The authority provides a free pre-hospital care both from the primary scene to a health facility or for inter-facility transfers. Under the authority, there is one central dispatch center for fire and pre-hospital services, eight ambulance stations, increasing number of ambulances and emergency medical technicians (EMT). In addition, a massive expansion of EMS is anticipated across Ethiopia. However, prior studies in other African countries have demonstrated that despite implementing an EMS system, public access remains hampered for a variety of reasons, including patient knowledge, beliefs, and culture.

In an effort to improve the pre-hospital care, understanding trends in EMS use by the public, including barriers and facilitators to pre-hospital care utilization, is important for the ultimate success of EMS in Addis Ababa. To the best knowledge of the investigators, no such prior EMS research has been done in Addis Ababa.

## Objective

The primary objective of the study was to assess the proportion of patients who used EMS, stratified by time-sensitive traumatic and medical emergencies. The secondary objectives were to quantitatively and qualitatively understand the barriers to EMS utilization in Addis Ababa.

## Methodology

### Study design and setting

A cross sectional quantitative and qualitative mixed study design was conducted in Addis Ababa. The city is the capital of Ethiopia with a population of more than 4.6 million people. The majority the population is less than 30 years of age. The common languages spoken in the city include Amharic (71.0%), Oromiffa (10.7%), Gurage (8.37%), and Tigringa (3.60%). In addition Oromiffa is the major language spoken in rural Addis Ababa and surrounding zones. Patients visiting emergency centers of selected Addis Ababa hospitals with time sensitive disease and trauma were included in the study. The city has 11 public hospitals, five of which were specifically selected for inclusion in this study (St. Paul’s hospitals millennium medical college (SPHMMC), Tikur Ambassa Specialized hospital (TASH), All African leprosy and tuberculosis rehabilitation and training (ALERT) Hospital, Tirunesh Beijing Hospital, and Minilik II hospital). The selected hospitals are tertiary care public hospitals and provide advanced trauma care. In addition, the hospitals are located in different directions and in the gateways of the city. These parameters for hospital selection allowed for a patient sample with varying socio economic, clinical and demographic backgrounds and minimized double counting.

### Sampling

The study period was for one month in March of 2017. The assumption was made that there are no significant differences in emergency trends and ambulance use in Addis Ababa based on month. All consecutive emergency patients who arrived directly from the scene in the study month and met inclusion criteria were included. The inclusion criteria were those patients who sustained severe trauma (labeled red or orange by South Africa Triage scale) and illnesses with time sensitive conditions (acute respiratory distress, stroke, and chest pain). The exclusion criteria included Laboring mothers, critically ill patients with no reliable surrogate, and cases of inter-facility transfer from another health care facility.

### Data collection procedures

A modified standard survey instrument was used [7]. The questionnaire included demographics, previous ambulance use, how the patient accessed an ambulance, length of time to access the ambulance, care given at the scene, care given during transportation, triage category, and parameters for knowledge and perception assessment. In addition an in-depth interview was conducted on 30 purposively selected participants. Before initiating data collection, the questionnaire was pre-tested on patients and individuals who accompanied them in all of selected hospitals. Pre-testing assessed the applicability of the survey instrument and facilitated improvement of the format and wording. Analysis of data from a similar study in Gabon [8] and our pre-test results indicated that responses were acceptably similar whether interviewing the patient or a relative who was at the scene. Accordingly, a patient was selected for an interview if he/she could provide history or a companion of the patient was able to provide the full interview. Off duty nurses working in emergency rooms of the study hospitals were recruited as data collectors. Ten data collectors, two for each hospital were trained in data collection. The training was in two sessions, one day a week, for two weeks prior to the data collection time.

### Data management and analysis

During the data collection, the questionnaires were checked for completeness and quality by supervisors and lead investigators. Data was collected during March 2017 and then the lead investigators cleaned, coded, entered and analyzed results using SPSS version 20. Descriptive statistics and logistic regression were done for quantitative data. An analytic model was developed to assess the effect of independent variables on the primary outcome variable (ambulance use). Independent variables included sex, age, language spoken by responder, distance from scene to hospital, car ownership, patient accompaniment, type of emergency, scene of emergency, belief of importance in ambulances, believing ambulance is faster than taxi, previous ambulance use, attitude towards quality, and educational status, all of which were assessed as part of the survey. To explore the relationship between independent variables and the outcome variable, descriptive cross tabs with chi-square analysis were performed. Variables were selected according to previous literature and the expert opinion of the authors. Variables that were found to be significant in bivariate analysis at the 0.1 level were entered into a multivariate model. A qualitative data from a total of 30 interviewees, 6 from each hospital, was translated, transcribed arranged thematically by the lead investigators.

### Ethical considerations

A written ethical clearance regarding the study was obtained from St. Paul Hospital millennium medical college institutional review board (IRB). Permission was received from the participating hospitals’ emergency departments. Informed consent was directly obtained from study participants. For unconscious patients, their surrogate was asked to provide consent and for minors (defined as children less than 18 years of age); their guardians were asked to consent. Autonomy and confidentiality were preserved during the study and during dissemination of the results. Qualitative data was coded and kept safe with the lead investigators and removed from the audio data collection tool.

## Results

A total of 455 participants were approached and 429 of them completed the survey, with a non- response rate of 5.1%. Of the participants, 122(26.6%) were recruited from SPHMMC, 118(26%) from TASH, 80(17.6%) from Tirunesh Beijing, 79(17.7%) from Minillik II hospital and 56(12.3%) from ALERT hospital. Of the 429 participants who completed the survey 83(19.3%) of interviewees were patients, 323(75.3%) were relatives of the patients and 23(5.4%) of the respondents were policemen who brought the patient to the hospital.

### Demographics of study participants

A large majority of respondents were male (*n* = 297, 69.2%) and the mean age of all patients was 33.8 years (SD, 10), with higher number of respondents were between 31 and 50 years (*n* = 210, 49.0%). Most of them were self-employed (*n* = 137, 31.9%) and majority have no car (*n* = 389, 90.7%). In regards to residency, most of the respondents resided in Addis for more than 25 years (*n* = 166, 38.7%) (Table 1).

**Table 1:** Demographic data of survey participants, Addis Ababa, Ethiopia (*N* = 429)

		Number of Patients (*n* = 429)	Percentage
Sex	Male	297	69.2
	Female	132	30.8
Age	18–30 years	192	44.8
	31–50 years	210	49.0
	> 50 years	27	6.3
Occupation	Student	35	8.2
	House wife	52	12.1
	Government worker	139	32.4
	Nongovernment organization	6	1.4
	Self employed	137	31.9
	Retired	9	2.1
	Unemployed	14	3.3
	Daily laborer	30	7.0
	Other	7	1.6
Language	Amharic	353	82.3
	Oromifa	42	9.8
	Tigrigna	29	6.8
	Others	5	1.2
Educational status	Primary	67	15.6
	Secondary	126	29.4
	Diploma	107	24.9
	Degree	98	22.8
	Post graduate	14	3.3
	Informal education	11	2.6
	Other	6	1.4
Length of residency in Addis	< 1 year	5	1.2
	2 to< 5 year	54	12.6
	5 to < 10 year	75	17.5
	10 to 25 years	129	30.1
	> 25 years	166	38.7
Marital status	Single	126	29.4
	Engaged	17	4.0
	Married	276	64.3
	Widowed	1	.2
	Divorced	9	2.1
Car ownership	Yes	40	9.3
	No	389	90.7

### Emergency medical service use

A significantly lower proportion of patients (*n* = 87, 20.3%) used an ambulance for their current emergency condition; the majority of patients used a taxi or private car (*n* = 326, 74.2%). Patients were brought to hospital mainly accompanied by family members (*n* = 329, 76.7%). The most common emergency scene was the patient’s residence (222, 52.8%), followed by road-side (n = 159, 37.1%). A larger proportion of trauma patients were extricated and moved from the site of trauma by a by stander (*n* = 116, 58%), followed by police (*n* = 48, 24%). Amongst the ambulance utilized groups, the median waiting time for ambulance arrival was 21 min (IQR 17). Eighty-one (93.1%) of the ambulance transported patients were able to name one ambulance call number (Table 2).

**Table 2:** Modes of transportation for emergency condition among survey patients (*N* = 429)

Characteristics		Mode of transport				Total Number (*n* = 429)
		Ambulance		Other		
		Number	Percentage	Number	Percentage	
Type of emergency	Illness	37	16.2	192	83.8	229
	Trauma	50	25.0	150	75.0	200
Patient age	13–18 years	5	18.5	22	81.5	27
	19–30 years	34	24.6	104	75.4	138
	31–50 years	29	18.8	125	81.2	154
	> 50 years	19	17.3	91	82.7	110
Patient accompaniment	unaccompanied	3	50.0	3	50.0	6
	Police	12	42.9	16	57.1	28
	Bystander	7	19.4	29	80.6	36
	Family/Relative	61	18.5	268	81.5	329
	Car driver	0	0.0	13	100	13
	Other	4	23.5	13	76.5	17
Means of extrication from the trauma site	Bystander	26	22.4	90	77.6	116
	Police	20	41.7	28	58.3	48
	Patient	2	25.0	6	75.0	8
	Ambulance Crew	3	100	0	0.0	3
	Other	2	8.0	23	92.0	25
Emergency scene	Home	35	15.8	187	84.2	222
	Work	5	21.7	18	78.3	23
	School	0	0.0	4	100	4
	Road side	43	27.0	116	73.0	159
	Sport/recreation area	3	15.8	16	84.2	19
	Other	1	50.0	1	50.0	2

Multivariate logistic regression analysis was done to assess the factors determining the dependent variable (Ambulance use). The factors in the model included sex, age, language spoken by responder, distance from scene to hospital, car ownership, patient accompaniment, type of emergency, scene of emergency, believing ambulance is faster than taxi, previous ambulance use, and educational status. Significant association was found in language, patient companion, and previous ambulance use (Table 3). Patient companion was categorized as police man, bystander and family /relatives. Patients who were companied by police (OR = 1.53) were positively associated with ambulance use. Language spoken by respondents was categorized as Amharic and non-Amharic speakers. Failure to speak Amharic was negatively associated with ambulance use *P* = 0.001. Previous ambulance use (P = 0.001) was positively associated to current ambulance use. Believing an ambulance is faster than a taxi or private car was positively associated with ambulance use, but the data were not statistically significant (*P* = 0.77).

**Table 3:** Factors affecting ambulance use: Logistic regression analysis result, Addis Ababa, Ethiopia

	OR	95% C.I.		*P* value
		Lower	Upper	
Language spoken by responder (non-Amharic speaking)	0.47	0.31	0.71	0.001
patient accompaniment (by Police)	1.53	1.11	2.12	0.01
Previous ambulance use	3.23	1.68	6.18	0.001
Believing ambulance is Faster than taxi/ private car	2.0	1.0	5.0	.077

### Knowledge and perception of emergency medical service use

Almost all of the participants (96.3%) believed ambulance was important for their emergency condition. The two common mentioned benefits from ambulance use were treatment during transport (*n* = 177, 42.4%) and faster transfer to hospital (*n* = 165, 40.4%). A higher proportion of participants believed ambulances are safer (n = 341, 79.5%) and faster (*n* = 298, 69.5%) than taxi or private car. The majority also believe there is high quality care in ambulances (*n* = 300, 69.9%). However, a significantly high proportion of participants perceived that there are not enough ambulances in Addis Ababa (*n* = 305, 71.1%). There is also significant discrepancy between the acceptable and actually waiting time. The median acceptable time to get the ambulance (according to respondent’s perception) was 16 min but actually perceived ambulance waiting time was 40 min. See Table 4 for more detail.

**Table 4:** Knowledge and perception of emergency medical service use, Addis Ababa, Ethiopia

			Frequency	Percentage
Availability (*n* = 429)	Perception of enough ambulances	Yes	124	28.9
		No	305	71.1
	Ever made ambulance call	Yes	156	36.4
		No	273	63.6
	Ever used an ambulance	Yes	74	17.2
		No	355	82.8
Accessibility	Time expected to get ambulance during rush hour (median, 25,75 percentile)	40.00(25.00,60.00)	NA	NA
	Time expected to get ambulance in non-rush hours (median, 25,75 percentile)	30.00(15.00, 40.00)	NA	NA
	Acceptable duration to get ambulance at any time (median, 25,75 percentile)	16.00(10.00,30.00)	NA	NA
	Can name one ambulance number (n = 429)	Yes	229	53.4
		No	200	46.6
	Can name 939 as an ambulance number (n = 229)	Yes	179	78.2
		No	50	21.8
	Perception of getting an ambulance on call 939 (*n* = 429)	Yes	222	51.7
		No	207	48.2
Accommodation (n = 429)	Perception that an ambulance is important for patient condition	Yes	413	96.3
		No	16	3.7
	Importance of ambulance	Treatment during transport	177	42.4
		Onsite patient treatment	35	7.8
		Fastest transportation means	165	40.4
		patient transfer	36	8.8
Affordability (n = 429)	Knowledge of free ambulance	Yes	331	77.2
		No	98	22.8
Acceptability (n = 429)	Perception of high quality care in ambulance	Yes	300	69.9
		No	117	27.3
		I do not know	12	2.8
	Perception that taxi is safer than ambulance	Yes	88	20.5
		No	341	79.5
	Perception that taxi is faster than ambulance	Yes	131	30.5
		No	298	69.5

A slightly higher proportion of interviewees named at least one ambulance number (*n* = 229, 53.4%), and the majority of them recalled 939 as the emergency ambulance number (*n* = 179, 78.2%). In regards to the source of information for ambulance numbers, a majority of the respondents were informed via radio (*n* = 128, 56.3%), followed by television (*n* = 54, 23.9%). Most participants knew there was a free ambulance service in Addis Ababa (*n* = 311, 71.2%) but almost half of the participants did not believe they could get the ambulance by calling the toll free ambulance number 939 (*n* = 202, 48.2%).

During in-depth interviews regarding the barriers to use ambulance, the majority of interviewees confirmed the findings of the quantitative results. Long arrival time for ambulance called during emergencies, not enough distribution of ambulance stations, and difficulty of accessing the phone were additionally emphasized. Most responded (*n* = 27, 90%) that if they can get to a phone, they are sure they will get the service. They were asked if the ambulances were misused in the city, for which most participants (*n* = 23, 77%) opined that, as far as their knowledge goes, ambulances were being used for only intended purposes. Only a few (*n* = 3, 10%) reported misuse other than for the intended purpose. See Table 5 below for selected quotes from the qualitative responses.

**Table 5:** Selected Quotas form in-depth interview of emergency medical service use in Addis Ababa, Ethiopia

Perceived use of ambulance in Addis Ababa	Perceived barrier to utilization
“ambulances are preferred for emergency patients appropriate transportation and for fast transport of patients” “ambulance is a care giver vehicle that arrive fast during accident” “are for the problem like fire and disease.” “I did not seen ambulances who are being used for other purpose” “ambulances should arrive fast while going to the patient” “more than 90% of ambulances are being used for intended use”	“In the city waiting ambulance is difficult due to over crowed of the roads and less distribution” “ambulances station distribution is not accessible” “I do not think ambulances are being used for the intended purpose only, like they carry coal” “ unavailability of road make difficult to use ambulance” “ambulance dispatches do not respond for the call.” “there is knowledge gap on their number and their use. There is also perceived inaccessibility.” “There are ambulance owner who are using for their own benefits using the name of ambulance care”

## Discussion

Only 20.3% of patients used an ambulance, and a significantly higher proportion arrived by taxi or private car (*n* = 326, 74.2%). Although there are no global standards for appropriate utilization rate for ambulances [9], the proportion of ambulance utilized patients were lower than expected. The study only looked at patients who were critically ill and hence ambulance use was expected to be higher. The percentage of use would have been even lower if we had included all patients. Non-Amharic speaking participants were amongst the least likely to utilize ambulance services. This could be because of the Amharic media of the call center, and hence there is a need to incorporate other languages like Oromiffa and Tigrigna in pre-hospital communication.

A similar study in Pakistan showed ambulance utilization for arrivals to the ED for all emergency patients to be 4.1% [10, 11], but a higher percentage of 30–67.3% was reported from India and developed nations [12, 13]. In these studies, the mean age of patients in the ambulance used group was significantly higher compared to the mean age of the non-ambulance group. But in this case and in a study from Ghana [7], younger patients are more likely to use ambulance. This may be due to overall young population of Addis Ababa.

Among the ambulance utilized groups, the median waiting time for ambulance arrival was 21 min (IQR 17). This is more than double the international recommended response time of eight minutes. Additionally, there was significant variation in the median acceptable time (according to respondent’s perception) to get the ambulance, 16 min, and actual perceived ambulance waiting time, 40 min. This was also emphasized in the qualitative study, and the time discrepancy may be the major barrier for utilization of ambulance services in case of emergency.

Patient residence was the most common emergency scene (222, 52.8%), followed by road side emergencies (*n* = 159, 37.1%), with a large proportion of trauma patients being extricated and moved from the site by a bystander (*n* = 116, 58%) followed by police (*n* = 48, 24%). Bystander training in Ethiopia is almost nonexistent. Research has shown that context appropriate bystander training has improved patient outcome with improvement of correct extrication, positioning, and control of hemorrhage [14]. These studies and the findings of our study may indicate an urgent need for implementation of context appropriate layman and policeman training on pre-hospital care.

There is favorable perception and ambulance knowledge; 53.4% of the participants named at least one ambulance number and the majority perceive that ambulances are important in emergencies and that there is high quality care in ambulances. The majority perceived that there are not enough ambulances or distribution of stations for ambulances in Addis Ababa and that under maintained roads lead to unacceptably higher waiting times. In a similar study in Accra, participants believed ambulances in Accra were insufficient though EMTs offered high quality care, but in the same study, in contrary to our finding, the majority (78.0%) believed taxis were faster than ambulances [7].

In a study done in Libreville, Gabon, factors such as lack of awareness, misperceptions, established alternatives, perceived response times and cost were reported as reason for underutilization of EMS [8]. In the Accra study, prior ambulance use and belief that ambulances are safer than taxi affected ambulance use [7]. Though most of the findings in the Libreville and Accra studies are in line with the results of this study, cost and misperception were not found to be barriers in this study. Improved training of bystanders also improves the detection, reporting, on-scene response, transit care and transfer to definitive care within the “golden hour” of trauma, yielding better outcomes [15]. In addition results indicate that there should be urgent action to coordinate ambulance services in Addis Ababa with improved quality and a more accessible distribution of ambulance stations. Community awareness on ambulances services needs to be expanded using radio and television.

### Limitations

The study was conducted only in urban public hospitals with trauma centers, making generalization to other settings difficult. It may also not represent actual community level utilization. Estimations of ambulance waiting time may have been effected by recall bias. In addition, the relatively small sample size of the study may have masked the effect of some factors contributing to ambulance utilization.

## Conclusion

Ambulance utilization level is low in Addis Ababa and emergency patients are instead being transported by taxi or private car. Perceived longer ambulance waiting time and language barriers may have contributed for low utilization. Findings of this study suggest an action to improve access by improving ambulance availability while simultaneously enhancing the public’s knowledge and perception of EMS in Addis Ababa.

## Abbreviations

ALERT: All African leprosy and tuberculosis rehabilitation and training
CI: Confidence interval
ED: Emergency department
EMS: Emergency medical services
OR: Odds ratio
RTI: Road traffic injury
SPHMMC: St. Paul’s Hospital Millennium Medical College
SPSS: Statistical Package for the Social Sciences
